# Scene Text Recognition Based on Bidirectional LSTM and Deep Neural Network

**DOI:** 10.1155/2021/2676780

**Published:** 2021-11-23

**Authors:** MVV Prasad Kantipudi, Sandeep Kumar, Ashish Kumar Jha

**Affiliations:** ^1^Department of E&TC, Symbiosis Institute of Technology, Symbiosis International (Deemed University), Pune 412115, India; ^2^Department of Computer Science and Engineering, Koneru Lakshmaiah Education Foundation, Vaddeswaram, AP, India; ^3^Nepal Engineering College, Kathmandu, Nepal

## Abstract

Deep learning is a subfield of artificial intelligence that allows the computer to adopt and learn some new rules. Deep learning algorithms can identify images, objects, observations, texts, and other structures. In recent years, scene text recognition has inspired many researchers from the computer vision community, and still, it needs improvement because of the poor performance of existing scene recognition algorithms. This research paper proposed a novel approach for scene text recognition that integrates bidirectional LSTM and deep convolution neural networks. In the proposed method, first, the contour of the image is identified and then it is fed into the CNN. CNN is used to generate the ordered sequence of the features from the contoured image. The sequence of features is now coded using the Bi-LSTM. Bi-LSTM is a handy tool for extracting the features from the sequence of words. Hence, this paper combines the two powerful mechanisms for extracting the features from the image, and contour-based input image makes the recognition process faster, which makes this technique better compared to existing methods. The results of the proposed methodology are evaluated on MSRATD 50 dataset, SVHN dataset, vehicle number plate dataset, SVT dataset, and random datasets, and the accuracy is 95.22%, 92.25%, 96.69%, 94.58%, and 98.12%, respectively. According to quantitative and qualitative analysis, this approach is more promising in terms of accuracy and precision rate.

## 1. Introduction

Understanding the visual scene is an active research area for the computer vision community. It needs enormous research in the field of computer vision and its subfields. Visual scene understanding includes the processing of both image and text, and it is always a difficult task to understand the scene and read the text written in the image. This research area is increasing gradually because it is helpful for many applications such as content-based image retrieval systems, assistance for blind people, automatic navigation systems in vehicles, and digitization of textbooks. OCR [1] is a traditional technique of recognizing the text from the documents, and the accuracy of this technique is good in the scanned documents; but when the same technique is applied to scene images, the performance of this method was not up to the mark [2]. The recognition of text from the scene needs special features because the character present in the scene may differ in size, shape, color, writing style, orientation, aspect ratio, quality of the image due to different lighting conditions, and blurred and complex background. These are the various challenges of text detection and text recognition. Generally, text detection identifies the location where exactly text is present in the image and creates a bounding box for each word or letter or line of text, and it also improves the accuracy of text recognition. The sample example of text detection is shown in the Figure 1.

Text recognition allows the computer to understand and predict the text in the given input scene image and convert it into the computer's understandable format. Text recognition is the most popular method for converting old printed documents into digitized forms. This process looks simple and more accessible because most of the image proceeding techniques follow the same. According to the literature survey, most of the text detection and recognition techniques are influenced by machine learning and deep learning techniques. Given the problems mentioned above and their solution, the main goal of this paper is to give a novel approach to text detection and text recognition based on deep neural networks and bidirectional LSTM. We proposed a scene text recognition method, and the proposed system is divided into three steps: in the first step, adaptive binarization technique is applied to the image so that the noise can be removed from the image, and it helps to extract the features from the blurred and complex background. In the second step, the contour detection technique is applied to the image, and it detects the meaningful area of the image, which makes the detection process easier and faster. In the third step, CNN-based architecture is designed in such a way that it can locate the text region and create a bounding box on each letter and also predict the characters. Here, CNN is combined with Bi-LSTM to make the classifier more powerful, and it is a handy tool for extracting the features from the sequence of words. This paper combines the two powerful mechanisms for extracting the features from the image and contour-based input image making the recognition process faster, which makes this technique better compared to existing methods. The complete detail of the proposed method is discussed in Section 3. The rest of the paper is structured as follows: Section 2 describes the related work. Section 3 discusses the proposed work.  Section 4 presents the experimental results and their comparison with existing methods.  Section 5 shows the conclusion and future scope.

## 2. Literature Work

Many researchers have worked on the various techniques of detection of the text in images. Some researchers explored the texture-based approach for locating the text information in the image and used the sliding window concept to analyze the unique texture present in the input image [3–7]. Some researchers focused on sparse-based text detection methods used for computer vision applications [8–12]. It is proposed by Zhao et al. [8]. These methods work to transform the image into edge maps. A further sliding window is used to extract the text patches present in the image, and then classification has been performed. Most researchers focus on deep learning-based methods for scene text detection and recognition, and a detailed comparative analysis has been done in Table 1.

A tremendous amount of work has been done in scene text recognition, and results are also satisfactory [27–32]. However, these algorithms cannot give better results if the background is complex, blurry, and has different lighting conditions. The computation cost is very high when the algorithms are applied to the real dataset. Therefore, it remains a challenge.

## 3. Proposed Work

The proposed method is divided into three steps: firstly, finding the contour of the image; secondly, the text detection is using CNN; and thirdly, the text recognition using combined RNN and Bi-LSTM. The detailed description is discussed further, and the flow chart of the proposed method is shown in Figure 2.

### 3.1. Contour Detection

The scene text recognition-based method is essential to identify the region where exactly text is present in the image. Rather than working on the whole image, only the object's boundary is sufficient for further processing. Considering the same, in the proposed method, the first contour of the image is identified [32]. Contour is used to find the boundary of the objects which is present in the image. These boundaries can be identified in different ways, such as finding the edges of the objects and finding the intensities of objects which are present in the image.

In the proposed method, we used the wireframe-based boundary detection method in which the whole image is traced using structuring elements, and the first pixel of the object is identified. This first pixel represents the component of the object. Identifying the first pixel in the image always depends on how the tracing has to begin in the input image.

The preferred direction of the tracing is the left most corner of the image and then towards the right direction of the image. The tracing of the image is continued until it will not find the contour of the whole image. Finally, all the boundaries of the objects are integrated, and the algorithm displays the contour of the image. The results of the contour detection are shown in Figure 3.

### 3.2. Text Detection Using CNN

The performance of any model always depends on the ability to discriminate the various features. An image-text can be arranged as a sequence of letters. A sequence of convolution and max-pooling layers are used to detect the text in an image. In the proposed method, four layers of CNN classify that the image's patch contains a character. The configuration of CNN is represented in Table 2 and Figure 4. First, the CNN classifier is trained with 62 classes in which 26 classes are used for uppercase letters, 26 classes are used for lower case letters, 10 classes are used for digits (0–9), and 1 for spacing. The image patches are directly classified as letters or digits; therefore, here, binary classifier is not required. The learned features are more specific and easy to discriminate from each other, making the learning process more accurate and speedy. The bounding box needs to be generated for each text present to detect the text in the image. The input image of this step is the contour image. There is a possibility that the input image can differ in size; therefore, to make it uniform, the size of the input image is 24 × 24, and each image is a greyscale image. First, the input image is padded from each side because if any character is near to the boundary of the image, then it can be detected through a sliding window. Using the sliding window, each row of the image is traced, NMS is performed to noise if it is present in the image, and the mean deviation and standard deviation of spacing are calculated. If the spacing value is lower than the threshold value, then it is considered that neighbour pixels are connected. Now, finally, the bounding box is identified for each character using a connected component analysis algorithm.

### 3.3. Scene Text Recognition Using Combined RNN and Bi-LSTM

This step is used to recognize the characters that are present in the image. Generally, the recognition system's performance depends on the segmentation techniques, but sometimes good segmentation will also lead to poor recognition because of noise, different lighting conditions, different sizes of text, rotation and illumination, etc. Deep learning-based methods are used, and in this paper, to overcome these problems, we combined RNN and LSTM to improve the recognition rate. The first features are extracted from the image. The CNN classifier is used for the sequential feature extraction from the image, and training is done for all 63 classes mentioned in Section 3.2. The feature extraction is done through the sliding window concept. The images which are already detected are the input for this step. The first padding of 12 pixels is done on the image, and the new image's size is now 24 × 94. For the partition of the padded image, a subwindow is used with size 24 × 24. Each portioned patch of the image is fed into the trained CNN, and this trained CNN extracts the features from the image with size 4 × 4 × 256 and 1000 features which are the output of the 4^th^ convolution layer and the first FC layer. These two feature vectors are combined, and it forms a one-dimensional feature vector of size 5096. PCA and normalization technique is applied to reduce the size of the feature vector. Now, the new feature vector is the size of 256-d, and these are the local and global features of the image. After extraction of local and global features from the image, the next step is feature labeling. For labeling of the feature, RNN is used in the proposed method. RNN is a unique neural network that can make use of past feature information, and it can also process the sequential inputs. To make the RNN more powerful, LSTM is combined here. LSTM has the capability of memorizing contextual information for a long time. LSTM consists of the memory cell and connection to itself and three gates that control the flow of information. The pictorial representation of the LSTM is shown in Figure 5.

*i*_*t*_ is the gate; *C*_*t*−1_ is the status at the last cell, and it is hidden; *f*_*t*_ is the forget gate; *H*_*t*_ is the final state of the latest *C*_*t*_; *W* is the weight of each connection; and *O*_*t*_ is the output gate. The following equations compute the values of the previous parameters:

(1) $$\begin{array}{c} i_{t}=\sigma \left(W_{xi}*X_{t}+W_{hi}H_{t-1}+W_{ci\circ }C_{t-1}+b_{i}\right),\\ f_{t}=\sigma \left(W_{xf}*X_{t}+W_{hf}H_{t-1}+W_{cf\circ }C_{t-1}+b_{f}\right),\\ C_{t}=f_{t\circ }C_{t-1}+i_{t\circ }\tanh\left(W_{xc}*X_{t}+W_{hc}H_{t-1}+b_{c}\right),\\ O_{t}=\sigma \left(W_{xo}*X_{t}+W_{ho}H_{t-1}+W_{co\circ }C_{t}+b_{o}\right),\\ H_{t}=O_{t\circ }\tanh\left(C_{t}\right). \end{array}$$

It is better to access the past and future contextual information to recognize the text string properly. Bi-LSTM consists of two hidden layers in which one hidden layer is used to process the features in the forward direction and the other is used to process the features in the backward direction. Both the hidden layers have produced the output using the same output layer. Bi-LSTM is applied recursively for each feature present in the feature sequence in the sequence labeling process. According to the computation (mentioned in the above equation), it takes input as the current state and neighborhood state; every time, *H*_*t*_ is updated. After that, a softmax layer is used to distribute the state of Bi-LSTM into a probability distribution for 62 classes. The one extra class is used for finding the space between two words. Finally, the feature sequence is transformed into the sequence of probability *P*.

Now, finally, the sequence of probability *P* must be transferred into a text string. In the proposed method, a CTC-based decoder is used for this purpose, and it is used for the classification of sequential text. For each time *t*, CTC calculates the probability distribution over the alphabet of possible characters, and it gives the characters which have the highest probability as output. The CTC object function is defined as follows:

(2) $$\begin{array}{c} O=-\sum_{\left(i_{s},t_{s}\right)\varepsilon S}\ln\;P\left(t_{s}|i_{s}\right). \end{array}$$

It is the negative log probability function of the network which correctly labels the training dataset. Here, *D* represents the training dataset which consists of input and target sequence, and it is represented by (*i*_*s*_, *t*_*s*_). Conditional probability is represented by *P*(*t*_*s*_*|i*_*s*_). The target *O* must be minimized, and it is equivalent to maximize the *P*(*t*_*s*_*|i*_*s*_). The object function is directly connected to the output of the Bi-LSTM layer, and it is defined as

(3) $$\begin{array}{c} P\left(i_{s}|t_{s}\right)=\sum_{\pi :B\left(\pi \right)=ts}P\left(\pi |p\right). \end{array}$$

The model is trained using gradient descent and backpropagation. In the above equation, *B* is used for removing the repeated and space labels. Suppose the sequence is *B* (*c*–*c*–*f*-), then the final output will be B(ccf). Once the model training is done, sequencing labeling aims to find the optimal path with max probability using Bi-LSTM.

## 4. Results

The experiments are performed on MSRATD 50 dataset, SVHN dataset, vehicle number plate dataset, SVT dataset, and random datasets to verify the performance of the proposed methodology. The experiments are performed on NVIDIA GTX 1650/60 Hz, 16 GB RAM, core-i7 10^th^ generation processor. 80% of the dataset images are used for training purposes to train and test the model, and 20% of the images are used for testing purposes. Hyperparameters used in the architecture are described in Table 2.

Existing methods are compared with the proposed method's accuracy. We used accuracy, recall, precision, and F1-score in evaluating the proposed method. The accuracy is defined as the percentage of correctly classified instances. It is used to calculate the proportion of true positive and true negative for multiclass classification problems. The formula for calculating accuracy, precision, recall, and F1-score is given as follows:

(4) $$\begin{array}{c} \text{accuracy}=\frac{\left(\text{TP}+\text{TN}\right)}{\left(\text{TP}+\text{TN}+\text{FP}+\text{FN}\right)},\\ \text{precision}=\frac{\text{TP}}{\left(\text{TP}+\text{FP}\right)},\\ \text{recall}=\frac{\text{TP}}{\left(\text{TP}+\text{FN}\right)},\\ F1_{\text{Score}}=2.\;\left(\frac{\text{precision}.\text{recall}}{\text{precision}+\text{recall}}\right). \end{array}$$

Here, TP = true positive, TN = true negative, FP = false positive, and FN = false negative.

### 4.1. MSRATD 50 Dataset

MSRA TD dataset is one of the benchmark datasets for text recognition, and this dataset contains 3000 images of 32 × 32 sizes. The dataset is challenging and noisy, and it contains English and Chinese text. The images in the dataset have blur and noisy background. The sample input images and the recognized text and its bounded box *x*-coordinate, *y*-coordinate, width, and height are listed in Figure 6. The proposed system had shown the accuracy of 95.22% and recall of 85.73%. The precision is 94.15%, and F-score is 87.09%. The metrics of the SVHN dataset are shown in Table 3.

### 4.2. SVHN Dataset

SVHN dataset (Street View House Numbers) is the dataset that contains 600,000 digital numbers captured from various angles from various houses of Google street view. All images are of size 32 × 32. The images are blurred and have images captured from a different angle. The obtained accuracy is 92.25%, and recall, precision, and F-score are, 79.03%, 92.49%, and 89.80%, respectively. The sample input images and the recognized text along with its bounded box *x*-coordinate, *y*-coordinate, width, and height are listed in Figure 7. The metrics of the SVHN dataset are shown in Table 4.

### 4.3. Vehicle Number Plate Dataset

We collected sample images from UFPR-ALPR dataset and tested them on our proposed method. The proposed method has shown an accuracy of 96.69%. The recall, precision, and F-score values are 93.11%, 86.77%, and 90.01%, respectively. The sample input images and the recognized text along with its bounded box *x*-coordinate, *y*-coordinate, width, and height are listed in Figure 8. The metrics of the SVHN dataset are shown in Table 5.

### 4.4. SVT Dataset

SVT dataset is one of the challenging datasets where the images were taken from Google street view. The images in the dataset are high variability and meager resolution. The proposed method has shown an accuracy of 94.58%. The recall, precision, and F-score values are 84027%, 91.86%, and 88.49%, respectively. The sample input images and the recognized text along with its bounded box *x*-coordinate, *y*-coordinate, width, and height are listed in Figure 9. The metrics of the SVT dataset are shown in Table 6. The dataset results are partially accurate as the images are the 3D projections of original image.

### 4.5. Random Dataset

We collected random text from the Internet to check the proposed method accuracy. The images were collected with a plain background and colored background. The accuracy of the proposed work is 98.12% as the samples contained the text and numbers without any noise in them. The obtained recall, precision, and F-score are 98.19%, 90.18%, and 97.07%, respectively. The sample input images and the recognized text along with its bounded box *x*-coordinate, *y-*coordinate, width, and height are listed in Figure 10. The metrics of the random dataset are shown in Table 7.

### 4.6. Comparison Analysis of the Proposed Work

We analyzed the proposed method on four benchmark datasets MSRA TD dataset, SVHN dataset, UFPR-ALPR dataset, SVT dataset, and random text collected from the Internet and phone camera. The datasets are challenging datasets in various aspects. MSRA TD dataset is a tiny dataset of street view door numbers dataset that contains only images of house numbers. The dataset contains a blurred dataset; the proposed system can recognize the number with 95.22% accuracy. The SVHN dataset is another challenging blurred dataset containing both text and numbers with different backgrounds and fonts, and the proposed system has shown an accuracy of 92.25%. The UFPR-ALPR is a vehicle number plate dataset with different backgrounds. The proposed system has shown an accuracy of 96.69%. We considered the SVT dataset, a Google street view dataset with heavy background fluctuations and unclear text with various fonts and 3D reflections. The proposed system has shown accurate results with 94.58% of accuracy. We collected random datasets from the Internet and few images captured from Samsung mobile phones with minimal resolution. The proposed system has shown an accuracy of 98.12%. The analysis is given in Table 8, and the corresponding graphs are plotted in Figure 11.

For some of the images, results are partially accurate. As we can see in Figure 12, the images which were captured from the long distance or the orientation of the image are different. In those cases, model is able to detect the text partially. Proposed work is compared with the existing state of art methods, and according to the analysis, precision and accuracy is improved. The average recognition rate of proposed methodology and the comparison with state of art methods are shown in the Table 9 and Figure 13.

## 5. Conclusion and Future Scope

This research paper proposed a novel approach for scene text recognition that integrates bidirectional LSTM and deep convolution neural networks. In the proposed method, first, the contour of the image is identified, and then, it is feed into the CNN. CNN is used to generate the ordered sequence of the features from the contoured image. The sequence of features now coded using the Bi-LSTM. Bi-LSTM is a handy tool for extracting the features from the sequence of words. Thus, this paper combines the two powerful mechanisms for extracting the features from the image and contour-based input image making the recognition process faster, which makes this technique better compared to existing methods. The proposed method is evaluated on four benchmark datasets MSRA TD dataset, SVHN dataset, UFPR-ALPR dataset, SVT dataset, and random text collected from the Internet and phone camera. According to the quantitative and qualitative analysis, this approach is more promising in terms of accuracy and precision rate. The datasets are challenging datasets in various aspects. The proposed method can able to detect the text from the different backgrounds, unclear text, blurred images, different font size, and different orientation. In future, a better approach can be introduced which can deal with heavy background fluctuations and different 3D reflections.

## Figures and Tables

**Figure 1:** Sample image of text-involved scenes of SVT dataset.

**Figure 2:** Block diagram of proposed work.

**Figure 3:** Original image and contour of the image on SVT dataset.

**Figure 4:** Block diagram of RCNN combined with Bi-LSTM.

**Figure 5:** Block diagram of LSTM.

**Figure 6:** Text recognition on MSRA dataset.

**Figure 7:** Text recognition on SVHN dataset.

**Figure 8:** Text recognition on vehicle number plates dataset.

**Figure 9:** Text recognition on SVT dataset.

**Figure 10:** Text recognition on random/self-dataset.

**Figure 11:** Overall text recognition on all dataset.

**Figure 12:** Incorrect text recognition on all dataset.

**Figure 13:** Comparative analysis of the proposed work with existing techniques.

**Table 1:** Literature study on existing methodology.

S. no.	Author & year	Methodology	Dataset	Performance
1	S. Yasser Arafat et al. [12], 2020	Faster RCNN + two stream deep neural network (TSDNN)	UPTI dataset	Avg. precision = 98%
				R. R. = 95.20%
2	Asghar Ali Chandio et al. [13], 2020	Multiscale and multilevel features	Chars74 K and ICDAR03 datasets	Precision = 90%
				Recall = 91%
				F-score = 91%
3	Yao Qin et al. [14], 2020	Faster RCNN + BLSTM	ICDAR 2015 datasets	Precision = 89.8%
				Recall = 84.3%
				F-score = 86.9%
4	Jheng-Long Wu et al. [15], 2020	BLSTM + CNN	Corpus dataset	Macro-F1 = 72%
				Micro-F1 = 71%
5	S. Yasser Arafat et al. [16], 2020	(AlexNet and Vgg16) + BLSTM	UPTI dataset	Accuracy = 97%
6	Sardar Jaf et al. [17], 2019	Recurrent neural network (RNN) + BLSTM	English web treebank universal dependencies dataset	Precision = 91.43%
				Recall = 94.52%
				F-score = 92.20%
7	M. A. Panhwar et al. [18], 2019	ANN	Self-dataset	Accuracy = 85%
8	Yen-Min Su et al. [19], 2019	Contour + morphological operation + ROI	ICDAR datasets	Accuracy = 93.44%
				Recall = 79.16%
				F-score = 85.71%
9	Ling-Qun Zuo Su et al. [20], 2019	CNN + BLSTM	SVT dataset, IIIT5K dataset, ICDAR 2003 and 2015 dataset	Accuracy = 95.96%
				Accuracy = 98%
				Accuracy = 98.2%
				Accuracy = 91%
10	Baoguang Shi et al. [21], 2017	CRNN	SVT dataset, IIIT5K dataset, ICDAR dataset	Accuracy = 97.5%
				Accuracy = 97.8%
				Accuracy = 98.7%
				Accuracy = 89.6%
11	Xiaohang Ren et al. [22], 2017	Text structure component detector (TSCD)	Ren's dataset, Zhou's dataset, Pan's dataset	Precision = 82%
				Recall = 72%
				F-score = 77%
12	Xiang Bai et al. [23], 2016	Bag of strokelets + HOG	SVT dataset, IIIT5K dataset, ICDAR 2003 dataset	Accuracy = 80.99%
				Accuracy = 85.6%
				Accuracy = 82.64%
13	Mingkun Yang et al. [24], 2021	CAPTCHA system	IIIT5K, SVT, IC03 IC13, IC15, SVTP CUTE	Accuracy = 92.9%, 89.6%, 92.5%, 92.2%, 76.8%, 80%, 77.1%
14	Anna Zhu et al. [25], 2021	Anchor selection-based region proposal network	ICDAR2013, ICDAR2015, and MSRA-TD500	Precision = 90.18%, 83.34%, 84.67%
				Recall = 91.16%, 79.99%, 80.37%
				F-score = 90.62%, 81.63%, 82.49%
15	ZiLing Hu et al. [26], 2021	Text contour attention text detector	ICDAR2015, CTW1500	Precision = 88.9%, 86.5%
				Recall = 85.2%, 80%
				F-score = 87%, 83.1%

**Table 2:** Hyperparameters used in the proposed work.

Parameter	Value
Epochs	50
Validation_split = 0.1	0.1
Drop out	0.2
Filters	16
Batch_size	64 × 64
Learning rate	0.00001

**Table 3:** Metrics of MSRATD 50 dataset.

Sr. No.	Parameters	Output
1	Precision	94.15
2	Recall	85.73
3	F-score	87.09
4	Accuracy	95.22

**Table 4:** Metrics of SVHN dataset.

S. no.	Parameters	Output
1	Precision	92.49
2	Recall	79.03
3	F-score	89.80
4	Accuracy	92.25

**Table 5:** Metrics of UFPR-ALPR dataset.

S. no.	Parameters	Output
1	Precision	93.11
2	Recall	86.77
3	F-score	90.01
4	Accuracy	96.69

**Table 6:** Metrics of SVT dataset.

S. no.	Parameters	Output
1	Precision	91.86
2	Recall	84.27
3	F-score	88.49
4	Accuracy	94.58

**Table 7:** Metrics of random/self-dataset.

S. no.	Parameters	Output
1	Precision	90.18
2	Recall	98.19
3	F-score	97.07
4	Accuracy	98.12

**Table 8:** Metrics of various datasets used in the proposed system.

S. no.	Parameters	MSRATD 50	UFPR-ALPR	SVHN	SVT	Random/self
1	Precision	94.15	93.11	92.49	91.86	90.18
2	Recall	85.73	86.77	79.03	84.27	98.19
3	F-score	87.09	90.01	89.80	88.49	97.07
4	Accuracy	95.22	96.69	92.25	94.58	98.12

**Table 9:** Metrics of various datasets used in the proposed system.

S. no.	Parameters	Ref. [22]	Ref. [19]	Ref. [18]	Ref. [14]	Proposed work (average)
1	Precision	82	—	91.43	90	92.15
2	Recall	72	79.16	94.52	91	83.50
3	F-score	77	85.71	92.20	91	88.56
4	Accuracy	—	93.44	—	—	93.83

## Data Availability

The data used to support the findings of this study are available from the corresponding author upon request.
